# An Effective Method for Detecting and Classifying Diabetic Retinopathy Lesions Based on Deep Learning

**DOI:** 10.1155/2021/9928899

**Published:** 2021-05-31

**Authors:** Abdüssamed Erciyas, Necaattin Barışçı

**Affiliations:** Department of Computer Engineering, Gazi University, Ankara, Turkey

## Abstract

Diabetic retinopathy occurs as a result of the harmful effects of diabetes on the eyes. Diabetic retinopathy is also a disease that should be diagnosed early. If not treated early, vision loss may occur. It is estimated that one third of more than half a million diabetic patients will have diabetic retinopathy by the 22nd century. Many effective methods have been proposed for disease detection with deep learning. In this study, unlike other studies, a deep learning-based method has been proposed in which diabetic retinopathy lesions are detected automatically and independently of datasets, and the detected lesions are classified. In the first stage of the proposed method, a data pool is created by collecting diabetic retinopathy data from different datasets. With Faster RCNN, lesions are detected, and the region of interests are marked. The images obtained in the second stage are classified using the transfer learning and attention mechanism. The method tested in Kaggle and MESSIDOR datasets reached 99.1% and 100% ACC and 99.9% and 100% AUC, respectively. When the obtained results are compared with other results in the literature, it is seen that more successful results are obtained.

## 1. Introduction

Diabetes occurs as a result of insufficient production of insulin or insufficient use of produced insulin [1]. There are many organs damaged by diabetes. For example, diabetic nephropathy damaging kidney nephrons, diabetic neuropathy damaging brain neurons, and diabetic retinopathy damaging eye retina can be given [2]. Diabetic retinopathy (DR) is a type of type II diabetes in which the retina of the eye is damaged and if left untreated, the disease can progress to vision loss [3]. DR's effect on the eye is often blurred or complete loss of vision [4]. The risk of blindness in diabetic patients is many times higher than in a healthy person. Therefore, DR is one of the leading causes of blindness in the world between the ages of 20 and 65 [5]. The World Health Organization (WHO) stated that up to half a million people are at risk of DR [6]. The economies of low- and middle-income countries suffer seriously from diabetes. By 2040, it is estimated that 33% of 600 million diabetic patients worldwide will have diabetic retinopathy [7].

Deep learning (DL) started with the work of LeCun et al. [8]. DL's popularity began in 1998 with the success of the convolutional neural network (CNN), a DL method used by his student Krizhevsky [9] at the 2012 ImageNet [10] competition. In the years after AlexNet on ImageNet, GoogleNet [11], InceptionV3 [12], VGGNet [13], ResNet [14], and DenseNet [15], networks were developed, and more successful results were achieved. Improvements in GPU hardware have a great impact on the success here. Because as the depth increases in the developed networks, the number of trained parameters increases in direct proportion. While the number of parameters in GoogleNet is 6.8 M, there are 144 M parameters in the deeper VGG19. While CNN image classification was done, the CNN structure was modified for segmentation and object detection in the image. Region-based CNN (RCNN) [16], Fast RCNN [17, 18], Faster RCNN [19], Single Shot multiBox Detector (SSD) [20] and You Only Look Once (YOLO) [21, 22] appeared with this change. Experts believe that deep learning will facilitate medical studies in the coming years of medicine. The successes obtained in the works [23–30] on the subject support this idea; it is about the improvement, classification, segmentation, and detection of medical images and related to the images and taking vital precautions. Moreover, Limwattanayingyong et al. showed that DL was more successful when they compared sight-threatening DR (STDR) screening with educated human grading and DL grading [31].

When the studies about DR classification in the literature were examined in detail, each study performed a preprocessing stage before training the network with CNN. The reason for this is that the lesions do not have a certain shape or form and are scattered in the image. This causes classification errors by reducing the clarity of the lesions in the image. These preprocessing phases were generally traditional image processing methods. Also, each study focused on operations for a particular dataset, and different methods were used for each dataset. This is because the grading system of each dataset is different. In this study, we proposed the 2-stage method that detecting independent from the dataset and classifying diabetic retinopathy lesions, completely based on deep learning. In the first stage, we created a pool of selected DR datasets and trained with Faster RCNN. We automatically determined the lesion region of interests in the images without any special process for the images in different DR datasets and prepared a pretrained model for the classification process, which is the second stage of the work. We completed the classification process by training images with the attention mechanism we added to pretrained ImageNet models.

In the second part of the work, literature research was made, and DR features, related studies, and results were mentioned. In the third chapter, features of the proposed method used datasets, and DL methods used were mentioned. In the fourth chapter, the results obtained with the proposed method and the comparison of the results in the literature were mentioned. In the fifth and last section, information was given about the success, effects, and future works of the method.

## 2. Literature Review

### 2.1. Diabetic Retinopathy Datasets

There are many datasets belonging to DR in open access. Some of these are MESSIDOR [32], DIARETDB [33], IDRiD [34], and Kaggle 2015 DR Competition Dataset [35]. These datasets has been reviewed and graded by ophthalmologists. Each dataset can be used in a different grading system. For example, DR levels were graded from 0 to 4 in Kaggle, while in MESSIDOR, they were graded from 0 to 3. The MESSIDOR dataset contains 1200 images classified into 4 levels [36]. MESSIDOR was published in 2008 by Criann [37].

DIARETDB consists of 219 retinal images containing 25 healthy and 194 with DR symptoms. Images were classified as exudate (soft and hard), spots (red), and bleeding. The detected lesions were expressed in 5 different degrees with 0.25 intervals between 0 and 1. Kaggle dataset images were shared with an award-winning DR determination contest. Approximately, 90,000 right and left eye retinal images were reserved for the test of approximately 40% and 60% of the training set. Images were graded in five different classes according to the ETDRS [38] grading method. IDRiD is a dataset with DR lesions created in India. The dataset presented for ME detection classified DR in five levels according to the ETDRS grading method. The dataset contains 516 images (413 training sets, 103 test sets) [39].

### 2.2. Diabetic Retinopathy Symptoms

*Microaneurysms* (MA): these are deformations of the blood vessel walls of 1-3 pixels in images [40, 41].

*Bleeding/hemorrhages* (HM): bleeding/hemorrhages is a blood leaking from damaged capillaries [40, 42].

*Exudates/exudates* (EX): when blood leaks more through capillaries, it causes exudates that are usually yellow in the retina [43].

*Macular edema (*ME): it occurs when there is leakage from the vessels around the macula [44].

*Neovascularization* (NV): it occurs when veins grow into the vitreous [45].

Figure 1 shows the EX, HM, optic disc (OD), and macula in the DR retina. The OD is the reference point for DR detection [45–47].

### 2.3. Performance Metrics

The confusion matrix in Figure 2 shows the predicted number of outcomes for 2 classes (0 and 1). Accordingly, when the classification value is 1 and the obtained value is 1 then true positive (TP); else then false negative (FN) is obtained. When the classification value is 0 and the obtained value is 0 then true negative (TN); else then false positive (FP) is obtained.

Accordingly, performance metrics can be calculated with the following equations:

(1) $$\begin{array}{c} \text{Sensitivity}=\text{ TP Rate }\left(\text{TPR}\right)=\frac{\text{TP}}{\text{FN}+\text{TP}}, \end{array}$$

(2) $$\begin{array}{c} \text{Specificity }\left(\text{SPE}\right)=\frac{\text{TN}}{\text{FP}+\text{TN},} \end{array}$$

(3) $$\begin{array}{c} \text{Accuracy }\left(\text{ACC}\right)=\frac{\text{TN}+\text{TP}}{\text{FP}+\text{FN}+\text{TP}+\text{TN}}, \end{array}$$

(4) $$\begin{array}{c} \text{FP Rate }\left(\text{FPR}\right)=1-\text{SPE}, \end{array}$$

AUC (area under curve) is the area under the receiver operator characteristics (ROC) curve obtained with the change rates of FPR and TPR.

## 3. Related Works

There have been 747 studies on about DR in the literature [48]. In this section, studies on DR detection with deep learning are examined. Some of the studies created their own CNN models and used end-to-end learning (EE), while others used transfer learning (TL) using pretrained models available on ImageNet. In the studies, optic disc localization, lesion detection, and fundus classification procedures were performed on the DR images. Most of the studies used the MESSIDOR dataset. In end-to-end training, there are studies that create their own special models such as Zoom, ZFNet, and SI2DRNet.

The authors in [49] developed the ZFNet based on the Faster R-CNN in their work on the localization of the optical disc using a Hessian matrix. This study was conducted using the MESSIDOR dataset. Alghamdi et al. [50] first classified the images as OD or non-OD with the CNN they developed. Detected OD locations were classified by the second CNN module as normal, suspect, or abnormal. The MESSIDOR dataset was used in this study. In [51], the authors made changes before the last FC layer of the VGG model to find the OD, thresholding the probability map and obtaining the center of gravity of the pixels. This study was conducted using the MESSIDOR dataset. The authors in [52] developed a controlled CNN model to classify the ME lesion type. This study was conducted using the MESSIDOR dataset. In [53], HM is detected, and a 41-pixel square image containing HM was extracted from the original image. The resulting image was classified and labeled according to the number of HM removed. It was then given to the CNN network for training. The method was tested on a Kaggle and MESSIDOR datasets using a 10-layer CNN model. The authors in [54] used TL to determine DR in 1748 samples from the MESSIDOR dataset and DR in 9963 samples from the EyePACS dataset. Each image was graded 3 to 7 times by ophthalmologists. In [55], they created a CNN model by extracting rare local features with the structure they call Bag of Visual Words (BoVW) and Speed-Up Robust Properties (SURF). This study was conducted using the MESSIDOR dataset. Gargeya and Leng [56] proposed a CNN for DR detection by modifying ResNet. They evaluated the method with MESSIDOR. The authors of [57] proposed a pretrained CNN model that includes the attention network and crop network to detect suspicious patch sites called Zoom for DR detection. The management was developed using the MESSIDOR dataset. The authors in [58] created SI2DRNet-v1 by scaling the kernel size from 3 × 3 to 5 × 5 after each pooling layer in CNN. MESSIDOR was used in the model. The author in [59] developed a method for localizing blood vessels and a pretreatment for bound component analysis. Linear separation analysis was then used to reduce dimensionality. SVM was used for classification in this method. Kaggle dataset was used in this study. Quellec et al. [60] developed a CNN model to detect DR lesions. Heat maps created by this method were not optimized for diagnosis. In this study, Kaggle dataset was used. The authors of [61], proposed a method for EX detection using the LeNet model. They dismissed the EX zones and gave them input to the LeNet network for training. They made data replication before the training. The work was developed using the Kaggle dataset. In [62], the authors dealt with overfitting and skewed datasets in DR detection. They used data amplification to train the CNN model, which consists of 13 layers. Kaggle dataset was used in this study. In the work of Jinfeng et al.'s [63], an ensemble technique and two deep CNN models were proposed to detect all stages of DR using balanced and unbalanced datasets. First, they created 3 sub-datasets by dividing the Kaggle dataset into 3 parts. In the first model, they trained 3 datasets separately with DenseNet-121 and ensembled their results. In the second model, they trained 3 dataset separately with DenseNet-121, ResNet50 and Inception-V3, and ensembled their results. Then, the models were compared with each other.

When examined Table 1, the highest SEN value among the studies was 100, and Abramoff et al. have achieved. With the highest AUC of 99.0, Gulshan et al. have achieved. The highest ACC value of 99.4 was obtained by Xu et al. that have achieved.

When Table 2 was examined, the highest SEN and ACC values were 100 and 97.9, respectively, Mansour; with the AUC value of 95.5, Quellec et al. have achieved.

## 4. Materials and Methods

Based on the abovementioned shortcomings, a 2-stage method was proposed where all types of DR datasets could be trained using DL completely without preprocessing in traditional ways. If it is explained in more detail, since the use of CNN directly to classify DR is insufficient, the lesions should be clarified by preprocessing. In order to clarify the lesions, the region of interests(ROIs) of the lesion must be determined first. These regions can be made clear by using regional CNN with DL. As the regional CNN only detects objects, a CNN structure is needed for classification. For these reasons, Faster RCNN and CNN were used together, and a 2-stage method was developed. The first stage of the 2-stage method is the automatic detection of lesions and marking of the lesion ROIs, and the second stage is the classification of marked images with a model created by transfer learning and attention mechanism [64] (Figure 3).

### 4.1. Used DL Methods

CNN has a structure that learns these properties by determining the image properties. CNN consists of certain layers. The convolution layer (conv), as evident from its name, performs a filter operation by convolution of the input image with the kernel matrix. This layer reveals the details in the image. Pooling layer pools the input image with one of the maximum (max pool) or global average pooling (global avg pool-GAP) methods, resulting in an image smaller than the image size. The aim is to delete unnecessary details and make learning easier. The fully connected (FC/Dense) layer helps the classification process by image features at the end of the network. In this study, VGG [65], DenseNet [66], ResNet [67], Inception [68], NasNet [69], MobileNet [70], and InceptionResNet [71], which are pretrainig models in ImageNet, were used in order to make faster training (Figure 4).

Regional training in CNN is needed to focus on specific objects in the image and to identify and segment them. RCNN structures have been developed to perform these operations. In simple terms, RCNN returns the box corridors of the regions detected in the image and the classification results. The first developed RCNN [72] creates weak candidate regions, while Fast R-CNN [73] feeds an input image directly to the CNN and reshapes it to be passed to the FC layer by ROI pooling. Faster R-CNN [74] uses region proposal network (RPN) instead of the selective search algorithm, unlike Fast R-CNN (Figure 5).

## 5. Results and Discussion

### 5.1. Used Datasets

In the proposed 2-stage method, a total of 6400 image data were used, including 1200 from MESSIDOR, 5000 from Kaggle, and 100 from DIARETDB and IDRiD datasets. In the first stage, the dataset was divided into 400 training and 6000 tests to determine DR lesion ROIs. In the second stage, the marked 6000 data used for testing in the first stage were used. In the first stage, MESSIDOR, Kaggle, DIARETDB, and IDRiD datasets were used together to automatically detect lesions in different datasets. Since MESSIDOR and Kaggle datasets were used in the second phase, the test data of the first phase were used from these datasets. The training, test, and validation set of the data used in the two DL methods were given in detail in the relevant sections.  Table 3 shows the number of images in the datasets used in the proposed method and the number of training and test images used for each stage.

### 5.2. Detection of Lesions with Region-Based CNN

In this stage, EX and HM lesion ROIs on DR datasets were determined by training with Faster RCNN. For Faster RCNN training, a total of 400 data including EX and HM lesions from MESSIDOR, Kaggle, DIARETDB, and IDRiD datasets were selected randomly and labeled as EX and HM. 1100 remaining data from MESSIDOR and 4900 remaining data from Kaggle were used for the test of 6000 data in total. 80 of the 400 data used for training were used for validation. The purpose of using all datasets together in training is to diversify training and to automatically detect lesions for any dataset related to DR. With the trained model in the first step, the lesion ROIs were predicted in 6000 data as EX or HM and marked on the images as in Figure 6.

The marked images obtained in the first stage will be classified in the second stage by adding the attention layer to the pretrained ImageNet models. In the proposed model, the lesion ROIs were made clear so that the attention mechanism can work more efficiently.

When Figure 7 is analyzed, some images of proliterative DR are EX-weighted, and some are HM-weighted; some have only EXs while some have only HMs. With this information, it is seen that when grading DR, the density of the lesions is taken into account, not the type. Therefore, the ROIs in the lesion were displayed in one color, and the training phase was started as shown in Figure 8.

### 5.3. Classification of Detected Lesions

In this stage, the lesion ROIs detected in the DR images were classified by adding the mechanism of attention to the pretrained ImageNet CNN models. In this section, MESSIDOR and Kaggle datasets, which were used for testing at the first stage and marked on the image of the ROIs of the lesion, were used for DR classification. By ophthalmologists, the MESSIDOR dataset was divided into 4 classes (0-3) and the Kaggle dataset into 5 classes (0-4). The grading was not based on EX or HM lesions detected in the retina, but according to the intensity of any of the lesions in the retina, as seen in Figure 7. Therefore, lesion ROIs detected in the first stage are marked with the same color. During the training phase, the model was aimed to learn the lesion density by focusing on the marked lesion ROIs on the image and to give more accurate results. For this reason, the last layer of ImageNet models was changed with the mechanism of attention. The reason for the addition of the mechanism of attention is that the GAP added after pretrained models is simple because the prominent lesion ROIs are more important than others. Therefore, 4 convolution layers were added to unlock pixels in space before pooling. Then, the global weighted average pooling (GWAP) layer is created in which attention was multiplied by features and then divided by the sum of attention. Let {*x*_1_, *x*_2_, *x*_3_, ⋯., *x*_*n*_] be a finite nonempty array and the weights of the *x* in this array be {*w*_1_, *w*_2_, *w*_3_, ⋯., *w*_*n*_]. In this case, the weighted average ($\bar{x}$) of the array is calculated as follows [75]:

(5) $$\begin{array}{c} \bar{x}=\frac{\sum_{i=1}^{n}w_{i}x_{i}}{\sum_{i=1}^{n}w_{i}}. \end{array}$$

Let the dimensions of a 3D image be expressed by *x*, *y*, and *z*, respectively. Let IF (*x*, *y*, *z*) expresses image features, and AF (*x*, *y*, *z*) expresses attention features. GWAP in image pixels is calculated according to Equation (5) as follows:

(6) $$\begin{array}{c} \text{GWAP}\left(x,y,z\right)=\frac{\sum_{x}\left(\sum_{y}\text{A}\text{F}\left(x,y,z\right)\text{IF}\left(x,y,z\right)\right)}{\sum_{x}\left(\sum_{y}\text{A}\text{F}\left(x,y,z\right)\right)}. \end{array}$$

The Lambda layer was then added to the rescaling results by pixel count to include the missing values in the attention model. Finally, the model was obtained by adding 4 dense layers. The resulting model's hyper parameters were finely tuned for each ImageNet model individually to achieve the best results.

For classification, a total of 6000 data were used 1100 from MESSIDOR and 4900 from Kaggle whose lesion ROIs were marked on the image as a result of the test in the first stage. Since DR classes for MESSIDOR and Kaggle are not the same, they were evaluated by training and testing separately for the two datasets. In MESSIDOR, 880 data were used for training, and 220 data were used for testing. 176 of the 880 data used for training were used for validation. In Kaggle, we used 3920 data for training and 980 data for testing. 784 of 3920 data used for training were used for validation.

Figure 9 shows the ROC curve and AUC values drawn with the classification prediction results for the non-DR (DR level 0) and proliterative DR (MESSIDOR DR level 3, Kaggle DR level 4) classes in the MESSIDOR and Kaggle datasets in the second stage. While calculating the ROC curve, the average of each FPR and TPR prediction result formed with 980 test data in Kaggle and 220 test data in MESSIDOR reserved for the classification test was taken. Detailed performance criteria obtained as a result of the prediction in the second stage were explained in Tables 4 and 5.

Table 4 shows the results obtained by using the method with different pretrained models in the MESSIDOR dataset. According to the results, VGG16 and VGG19 achieved 100% value in all metrics. DenseNet201 achieved 100% in AUC.

Table 5 shows the results obtained by using the method with different pretrained models in the Kaggle dataset. According to the results, the best result in the SEN value was obtained with VGG16 with 99.1%, and the best results in the AUC value with 99.9% in VGG16 and the best results in the ACC value with 99.1% were obtained in VGG16 and VGG19.

Figure 10 shows the prediction results of marked DR images selected randomly and in different classes, obtained with the test data of the trained model using VGG16 and MESSIDOR dataset in the proposed method. The figure also shows the attention map obtained in the attention layer.

In Table 6, the results obtained in the studies that made the MESSIDOR dataset fundus classification were compared with our proposed study. Accordingly, our method achieved a better result than other methods in all metrics.

In Table 7, the results obtained in studies developed with the Kaggle dataset were compared with our proposed study. Accordingly, our method achieved a better result than other methods with 99.1% in ACC and 99.9% AUC values. With a sensitivity value of 100%, Mansour achieved better results than our method.

## 6. Conclusions

Deep learning gives successful results in disease detection. In this work, a deep learning-based method has been proposed in which diabetic retinopathy lesions were detected automatically and independently of datasets, and the detected lesions were classified. In the first stage, lesions were detected with the regional CNN, and the images obtained in the second stage were classified using the transfer learning and attention mechanism for diabetic retinopathy grading. When the method tested in Kaggle and Messidor datasets was evaluated, 99.1% and 100% ACC, and 99.9% and 100% AUC were obtained, respectively. When the obtained results were compared with other results in the literature, it was seen that more successful results were obtained.

In future studies, the algorithms using the method will be developed to use minimum system resources.

## Figures and Tables

**Figure 1:** EX, HM, optic disc (OD), and macula in the DR retina.

**Figure 2:** Confusion matrix.

**Figure 3:** Developed model structure.

**Figure 4:** Pretrained models: (a) VGG16, (b) VGG19, (c) ResNet, (d) Inception, (e) MobileNet, (f) InceptionResNet, (g) DenseNet, and (h) NasNet.

**Figure 5:** Faster RCNN architecture.

**Figure 6:** DR image, whose lesions are detected automatically with the trained model.

**Figure 7:** Proliterative DR images.

**Figure 8:** DR image with marked lesion region of interest.

**Figure 9:** AUC prediction values in the ROC curve for the model trained with VGG16 in the second stage for (a) MESSIDOR non-DR, (b) MESSIDOR proliterative DR, (c) Kaggle non-DR, and (d) Kaggle proliterative DR.

**Figure 10:** The predicted results of the training using the VGG16 model of the proposed method and the MESSIDOR dataset and the attention map obtained in the attention layer.

**Table 1:** Studies using MESSIDOR dataset and results.

Authors	Training type	Method	Process type	ACC	AUC	SEN
Zhang et al. [49]	ZFNet	TL	Optic disc localization	99.9		—
Alghamdi et al. [50]	CNN	EE	Optic disc localization	99.2	—	—
Xu et al. [51]	CNN	TL	Optic disc localization	99.4	—	—
Abràmoff et al. [52]	CNN	EE	Lesion detection	—	—	100
Grinsven et al. [53]	CNN	EE	Lesion detection	—	97.9	93.1
Gulshan et al. [54]	CNN	TL	Fundus classification	—	99.0	87.0
Costa and Campilho [55]	SURF + CNN	EE	Fundus classification	—	90.0	—
Gargeya and Leng [56]	CNN	EE	Fundus classification	—	94.0	—
Wang et al. [57]	Zoom	EE	Fundus classification	91.1	95.7	—
Chen et al. [58]	SI2DRNet	EE	Fundus classification	91.2	96.5	—

**Table 2:** Studies using Kaggle dataset and results.

Authors	Training type	Method	Process type	ACC	AUC	SEN
Grinsven et al. [53]	CNN	EE	Lesion detection	-	91.7	84.8
Mansour [59]	AlexNet + SVM	TL	Fundus classification	97.9	-	100
Quellec et al. [60]	CNN	EE	Fundus classification	-	95.5	-
Colas et al. [61]	CNN	EE	Fundus classification	-	94.6	96.2
Pratt et al. [62]	CNN	EE	Fundus classification	75.0	-	95.0
Jinfeng et al. [63]	CNN	TL	Fundus classification	80.3	-	-

**Table 3:** The number of images in datasets and the number of training and test images used for detection and classification.

Dataset	Total images	Number of images for detection stage training	Number of images for detection stage testing	Number of images for classification stage training	Number of images for classification stage testing
Kaggle	80,000	100	4900	3920	980
MESSIDOR	1200	100	1100	880	220
IDRiD	516	100	-	-	-
DIARETDB	219	100	-	-	-

**Table 4:** Results obtained by using MESSIDOR dataset and different pretrained models on the proposed method.

Model	TP	FN	TN	FP	ACC	AUC	SEN
VGG16	220	0	660	0	100	100	100
VGG19	220	0	660	0	100	100	100
DenseNet201	217	3	650	10	98.5	100	98.5
DenseNet121	195	25	658	2	96.9	97.6	88.6
DenseNet169	192	28	647	13	95.3	91.3	87.2
MOBILENET	192	28	574	86	87.0	94.5	87.2
NASNet	190	30	570	90	86.3	96.5	86.4
InceptionV3	200	20	593	67	90.1	94.2	90.1
InceptionResNetV2	192	28	574	86	87.0	87.0	87.2
Resnet50	186	34	560	100	84.7	89.8	84.5

**Table 5:** Results obtained by using Kaggle dataset and different pretrained models on the proposed method.

Model	TP	FN	TN	FP	ACC	AUC	SEN
VGG16	971	9	3887	33	99.1	99.9	99.1
VGG19	969	11	3889	31	99.1	99.7	98.9
DenseNet201	919	61	3865	55	97.6	98.6	93.8
DenseNet121	952	28	3894	26	98.9	99.6	97.1
DenseNet169	836	144	3811	109	94.8	98.5	85.3
MOBILENET	684	296	3630	290	88.0	92.6	69.8
NASNet	508	472	3496	424	81.7	83.8	51.8
InceptionV3	674	306	3683	237	88.9	92.3	68.8
InceptionResNetV2	540	440	3726	194	87.0	84.3	55.1
Resnet50	202	778	3142	778	68.2	82.4	20.6

**Table 6:** Comparison of studies conducted with the MESSIDOR dataset and the proposed study.

Authors	Training type	Method	Process type	ACC	AUC	SEN
Gulshan et al. [54]	CNN	TL	Fundus classification	—	99.0	87.0
Costa and Campilho [55]	SURF + CNN	EE	Fundus classification	—	90.0	—
Gargeya and Leng [56]	CNN	EE	Fundus classification	—	94.0	—
Wang et al. [57]	Zoom	EE	Fundus classification	91.1	95.7	—
Chen et al. [58]	SI2DRNet	EE	Fundus classification	91.2	96.5	—
Ours	Faster RCNN + CNN	TL	Fundus classification	100	100	100

**Table 7:** Comparison of studies conducted with the Kaggle dataset and the proposed study.

Authors	Training type	Method	Process type	ACC	AUC	SEN
Mansour [59]	AlexNet + SVM	TL	Fundus classification	97.9	-	100
Quellec et al. [60]	CNN	EE	Fundus classification	-	95.5	-
Colas et al. [61]	CNN	EE	Fundus classification	-	94.6	96.2
Pratt et al. [62]	CNN	EE	Fundus classification	75.0	-	95.0
Jinfeng et al. [63]	CNN	TL	Fundus classification	80.3	-	-
Ours	Faster RCNN + CNN	TL	Fundus classification	99.1	99.9	99.1

## Data Availability

Previously reported diabetic retinopathy datasets were used to support this study and are available at https://www.adcis.net/en/third-party/messidor/, https://www.kaggle.com/c/diabetic-retinopathy-detection/data, https://www.it.lut.fi/project/imageret/diaretdb0/, https://www.it.lut.fi/project/imageret/diaretdb1/, and https://ieee-dataport.org/open-access/indian-diabetic-retinopathy-image-dataset-idrid. These datasets are cited at relevant places within the text as references [32–35].
